# Duodenal Fibrosis Mimicking Neoplastic Obstructive Hepatopathy in the Setting of Lynch Syndrome

**DOI:** 10.7759/cureus.35679

**Published:** 2023-03-02

**Authors:** Oscar L Hernandez, Marwa Hussain, Zoilo K Suarez, Talwinder Nagi, Touqir Zahra

**Affiliations:** 1 Internal Medicine, Florida Atlantic University, Boca Raton, USA; 2 Medical School, Florida Atlantic University Charles E. Schmidt College of Medicine, Boca Raton, USA; 3 Internal Medicine, Florida Atlantic University Charles E. Schmidt College of Medicine, Boca Raton, USA

**Keywords:** endoscopic retrograde cholangiopancreatography (ercp), duodenal fibrosis, extrahepatic biliary obstruction, biliary obstruction, duodenal cancer, biliary diseases, lynch syndrome phenotype

## Abstract

Intestinal fibrosis is a rare complication of chronic inflammation resulting from various etiologies, including surgery, abdominal radiation, and inflammatory bowel disease. Consequences of intestinal fibrosis include intestinal dysmotility, malabsorption, and obstruction. Patients with Lynch syndrome are predisposed to developing intestinal adenocarcinoma including in the small intestines which typically require intra-abdominal procedures that expose them to fibrogenic triggers. Here, we present a rare case of duodenal fibrosis involving the sphincter of Oddi leading to malabsorption and gastrointestinal symptoms in a patient with Lynch syndrome requiring advanced endoscopy interventions.

## Introduction

Inflammation in response to injury can result in the regeneration of the damaged tissue or repair with the deposition of connective tissue components [1]. Fibrosis is a consequence of chronic inflammation that can induce myofibroblast stimulation with subsequent deposition of extracellular membrane components into affected tissues [2]. Certain insults are likely to induce a fibrotic response, such as radiation injury, in which 5-10% of patients receiving gastrointestinal (GI) radiation therapy develop obstructing fibrosis [3]. The development of radiation-induced GI fibrosis is a chronic process that can surface months to years after treatment [2]. Recurrent abdominal surgeries are another source of GI fibrosis, with 93% of patients having had multiple operations developing adhesions [4]. Surgical adhesions have multiple complications, including small bowel obstruction, the need for re-operation, and infertility in women [4]. Similarly, fibrosis is common in patients with inflammatory bowel disease due to the chronic inflammatory state. In patients, especially those with multiple comorbidities, many factors can lead to the development of GI fibrosis, portraying the potentially relentless sequence of intervention with possible recurrence of fibrosis. Here, we present a case of duodenal fibrosis presenting as a pancreaticobiliary obstruction in the setting of Lynch syndrome.

This case was presented as a poster at the American College of Gastroenterology Annual Scientific Meeting in 2021.

## Case presentation

A 61-year-old male with a past medical history of Lynch syndrome presented to an academic health center with a six-month history of weakness and progressively worsening fatigue associated with weight loss and chronic diarrhea. He described his diarrhea as pale and watery stools not associated with blood, of which he experienced three episodes per day. The patient denied associated abdominal pain, fevers, recent travel, or sick contacts. Given his previous history of Lynch syndrome, the patient had recurrent stage IV colorectal adenocarcinoma in both the small and large bowel complicated by previous pancreatic duct obstructions. His cancer was currently in remission post-chemotherapy, radiotherapy to the abdomen, and partial colectomy and subsequent distal duodenectomy, omentectomy, and primary duodenojejunostomy five years prior to presentation.

On physical examination, the patient was afebrile, normotensive, and in no acute distress. Physical examination findings included anicteric sclera, bradycardia with a heart rate of 35 beats per minute, and lungs that were clear to auscultation bilaterally. On abdominal examination, the patient’s abdomen was non-distended, with normoactive bowel sounds, and non-tympanic without tenderness. His skin was warm, pink, and without jaundice. Laboratory evaluation yielded a white blood cell count within normal limits and normocytic anemia with hemoglobin of 10.4 g/dL. Most concerning were his elevations in alkaline phosphatase, gamma-glutamyltransferase, and lipase at 1,217 IU/L, 995 IU/L, and 1,992 U/L, respectively (reference range: 44-147 IU/L, 5-40 U/L, and 0-160 U/L, respectively). Aspartate transaminase and alanine transaminase were 45 IU/L and 48 IU/L, respectively (reference range: 8-33 U/L and 4-36 U/L, respectively). Stool studies for his diarrhea lacked fecal leukocytes, ova, or parasites. Fecal elastase was low at less than 10 µg/g (reference range: >200 µg/g) with an elevated fecal calprotectin of 388 µg/g (reference range: >10-60 µg/mg).

A computed tomography (CT) scan of the abdomen and pelvis with contrast showed evidence of significant intrahepatic and bile duct dilation in addition to pancreatic duct dilation. The patterns of cholangiocyte, pancreatic injury, and fecal elastase results paired with the CT scan findings and his Lynch syndrome raised suspicions for a pancreaticobiliary obstruction secondary to a neoplastic recurrence with gallstone obstruction remaining within our differential diagnoses. A gastroenterologist with advanced endoscopy training was consulted for further evaluation, and an endoscopic retrograde cholangiopancreatography (ERCP) with endoscopic ultrasound (EUS) was performed. Endoscopy evaluation found numerous sessile polyps in the remnant of the duodenum with a track of fibrosis appearing to have fibrosis over the sphincter of Oddi. On visualization, his fibrosis appeared to directly extend from the site of the duodenojejunostomy as the point of origin.

ERCP was unsuccessful as the sphincterotomy with subsequent passage of a guide wire could not be achieved due to the extensiveness of the fibrosis overlying the sphincter of Oddi. Therefore, the decision was made to place a transgastric biliary drain to allow for the communication of obstructed common bile duct contents into the lumen of the stomach. Transgastric drain deployment would thus allow pancreaticobiliary excretions to enter into enteric transit. EUS was used to confirm common bile duct location through the gastric wall, and a transgastric biliary drain was deployed (Figure 1) with subsequent demonstration of the flow of obstructed contents into the stomach lumen upon stent deployment (Figure 2).

**Figure 1:** Deployment of a transgastric biliary drain through the gastric wall into the common bile duct.

**Figure 2:** Visible flow of accumulated biliary and pancreatic excretions through a transgastric drain demonstrating adequate placement.

Following the procedure, the patient was observed for two days while he was provided supportive care for his diarrhea, and his liver transaminases were trended. Over the observation period, the patient experienced relief in his diarrhea with the development of formed bowel movements and fewer than three bowel movements per day. His serum alkaline phosphatase and serum lipase levels demonstrated a downtrend to within normal limits. The fecal elastase level was checked on postoperative day two and showed improvement to 226 µg/g. The patient was discharged home on postoperative day three to follow up with his primary care physician and gastroenterologist as an outpatient. Upon re-evaluation three months postoperatively, the patient continued to report the resolution of his diarrhea and fatigue symptoms.

## Discussion

In evaluating our case, several points of interest arose when considering the pathophysiology contributing to our patient’s presentation of abdominal pain, diarrhea, and weight loss. Consideration of the etiology of the fibrosis noted in the patient’s duodenum was paramount to understanding what interventions were available. Duodenal fibrosis has been a rarely described complication in our review of the currently available literature. Although cases of duodenal fibrosis leading to intestinal dysmotility have been noted in several case reports, reports of primary fibrosis of the duodenum with secondary loss of pancreaticobiliary exocrine excretions have not been described [5,6].

Based on the distribution of the fibrosis surrounding the surgical anastomosis at the sight of the duodenojejunostomy, we can speculate that the primary source of fibrosis originated at this location. This fibrosis was noted to extend toward the proximal duodenal portion to involve the sphincter of Oddi, thus contributing to the loss of digestive excretions of the pancreaticobiliary system as excretions were unable to enter the enteric tract. A lack of enzymatic activity in the enteric tract including pancreatic lipase, amylase, and protease likely led to his subsequent weight loss and diarrhea symptoms as these enzymes are key for the digestion of fats, starches, and sugars, respectively [7]. This scenario is supported by the measured deficiency in pancreatic lipase in the patient’s stool sample early during his hospital course. Additionally, lack of bile excretion in the enteric tract, as demonstrated by the dilated biliary tree on initial CT imaging, likely further complicated his malabsorptive symptoms given the impaired absorption of dietary fats. Subsequent improvement of his symptoms following transgastric biliary drainage corresponded with improved stool pancreatic lipase levels to support malabsorption as the etiology of his symptoms.

Several factors are believed to have contributed to inducing fibrogenesis in the region of the duodenum seen in our patient. Rigby et al. have demonstrated the presence of fibrosis along intestinal anastomoses sites in previous studies [8]. Fibrosis along the surgical anastomosis site from his previous duodenojejunostomy appears to be the primary nidus of his fibrosis given the observed fibrosis distribution along his anastomosis site. Additionally, the patient’s abdominal radiation may have contributed to his progressing fibrosis as well. As noted by Haydont et al., abdominal radiation in the treatment of intra-abdominal malignancies can induce excess submucosal collagen deposition and subsequent fibrosis of the affected intestine [6]. The initial surgery with subsequent abdominal radiation following the patient’s postoperative course five years prior appears to have significantly contributed to his underlying fibrosis. Although Lynch syndrome has been known to cause chronic inflammation in the intestinal tract [9], no reports of gastrointestinal fibrosis in the absence of visible polyps have been found during our evaluation of the current literature. No polyps were noted during ERCP evaluation, and, therefore, we do not believe the fibrosis was a direct result of the patient’s Lynch syndrome, but rather a result of the interventions for the patient’s previous Lynch syndrome-associated small intestinal adenocarcinoma. Pharmacotherapy targeting fibrogenic cytokines exists for fibrosis-affecting tissues, such as cardiac, pulmonary, and hepatic tissues, although no current pharmacotherapies have been established for intestinal fibrosis [2]. Treatment to relieve the mechanical complications of intestinal fibrosis remains the mainstay of therapy including symptom-specific management. In this case, interventional gastroenterology techniques were used to bypass the sphincter of Oddi obstruction via the creation of a bypass conduit between the ampulla of Vater and the lumen of the stomach.

## Conclusions

In patients with surgical interventions or abdominal radiation presenting with non-specific abdominal symptoms and diarrhea, evaluation for intestinal fibrosis with endoscopy should be considered when other common causes are ruled out. Interventions to bypass obstructions and alleviate intestinal motility should be considered to improve morbidity in these patients. As seen in our case, the use of transgastric biliary stenting to circumvent cholestatic obstructions in the setting of duodenal fibrosis involving the sphincter of Oddi can provide reasonable benefit to these patients.
